This article has been retracted.

# An Analysis of Public Environment-Oriented Marxist Philosophy Content Dissemination

**DOI:** 10.1155/2022/7873226

**Published:** 2022-06-03

**Authors:** Jinming Guo, Haibo Hu

**Affiliations:** Northeast Normal University, Changchun 130024, China

## Abstract

Marxist philosophy has always been attached to the practice. In the new age, Marxist philosophy needs to solve many problems, such as ecological destruction, environmental pollution, international conflicts, and technical innovation, and improve the integration of the Marxist philosophy system with China's national conditions. The premise of change is practice, and the premise of practice is dissemination. Promoting the dissemination of Marxist philosophy is the cornerstone of solving the blind spot in the process of Marxist philosophy popularization. Because of the development of Internet technology, in order to ensure the validity of the uploaded videos related to Marxist philosophy on the platform, combining the research on human visual perception and the advantages of the long-term recurrent convolutional network (LRCN) model in video content recognition, an attention mechanism-based LRCN model is proposed, which simulates the attention characteristics of the human brain in the deep learning model, considers the video content globally, and makes the attention of the model fall in the effective area of the whole video. The experiment uses HMDB51, UCF101, and YouTube-8M data sets, and the results show that the LRCN model based on the attention mechanism proposed in this paper can effectively improve the accuracy of video content recognition, and it can converge quickly during training to improve the efficiency of model training.

## 1. Introduction

Marxist philosophy is the inevitable result of social development in the middle of the nineteenth century [1]. It is a theory about the proletariat and human liberation and realizes the unity of materialism and dialectics, materialistic natural view and historical view of materialism, and scientific and revolutionary view on the basis of scientific practice view, thus bringing about a revolutionary change in the history of philosophy. The establishment of Marxist philosophy is a revolutionary change in the history of philosophy [2–4]. The key reason why Marxist philosophy can launch a revolution shaking the history of human thought lies in that it scientifically solves the relationship between man and nature and between man and society based on the viewpoint of practice, thus realizing the unity of materialism and dialectics and materialist view of nature and materialist view of history. The viewpoint of practice is the primary and basic viewpoint of Marxist philosophy.

Philosophy is not equal to science. Philosophy may represent the views and theories of thinkers of a certain class, but it is not necessarily the true understanding of the objective world [5, 6]. However, philosophy and science are intrinsically related. Any science is to study and grasp a certain law as its own responsibility; philosophy is also with its unique perspective to study and grasp a certain law. As far as Marxist philosophy is concerned, it takes the relationship between man and the world as its object and reveals the general laws of the external world and the movement of human thinking through the reflection of natural science and social science [7–9]. In this sense, Marxist philosophy is science, with strict scientific nature. Marxist philosophy is not only integrated with practical activities but also closely linked with scientific activities, penetrating into the basic fields of natural and social sciences.

Marxist philosophy not only treats capitalist society with a critical attitude but also treats socialist society with a critical spirit, believing that socialist society is also a society in need of constant reform. Marxist philosophy not only treats other philosophical trends of thought critically but also treats its own theory in a critical spirit and carries on self-criticism [10]. Marxist philosophy never rests on its laurels and regards its own theory as the ultimate system of truth. History has proved that all systems of thought that claim to be the ultimate truth are doomed. Marxist philosophy will not repeat the mistakes of these thought systems. Its fundamental guarantee is that it consciously roots in practice; treats existing things and philosophical thoughts with a critical attitude; treats its theory with a critical spirit; develops its theory creatively with a strong sense of history and responsibility, according to the development of practice and scientific progress; and timely corrects some outdated viewpoints and conclusions proved by practice [11]. The critical nature of Marxist philosophy makes it a continuously developing theoretical system.

Marxist philosophy is inclusive and can be organically combined with the governing thought of any country in the world to continuously enrich and develop Marxist philosophy. It can be seen that Marxist philosophy has the characteristics of learning, guidance, publicity, and communication, but in fact, how to expand the dissemination of Marxist philosophy in the public environment is the issue we study. The age of we-media is the inevitable result of the development of science and technology, with distinct characteristics of the ages. We-media has become an important way for people to exchange information and has a profound impact on information transmission in various fields [12, 13]. In particular, it has a profound impact on the content, way, language, and environment of the dissemination of Marxist philosophy, which is embodied in the following aspects:

1. We-media has profoundly changed the communication system of Marxist philosophy. The emergence of we-media has enriched the communication form and mode of Marxism, enabling Marxist philosophy to spread through videos, images, and texts and further enhancing the influence of Marxist philosophy. In the practice teaching of Marxist philosophy, we-media can also be used to expand teaching content, enrich teaching means, and enhance the learning interest of the educated. Making full use of the advantages of we-media can further expand the communication channels of Marxist philosophy, especially the application of we-media such as Weibo and WeChat, closely combine the knowledge related to Marxist philosophy with social practical problems, and realize the dissemination of Marxist philosophy through the fan effect. At the same time, we should clearly see that the dissemination of traditional Marxist philosophy still has its own advantages, and we should combine traditional education methods with modern communication methods to jointly enhance the influence of Marxist philosophy.
2. The interactive advantages of we-media enhance the pertinence of Marxist philosophy communication. The main advantage of we-media lies in that it breaks the limitation of time and space and can realize interactive communication between people. One-to-one, one-to-many, many-to-many, and many-to-one communication can be realized through the we-media platform, which can effectively motivate ordinary people to participate in the dissemination of Marxist philosophy. Supported by big data and cloud computing, data analysis can specify different audiences' needs at different levels and make personalized communication plans according to different audiences' needs. In particular, people at different cultural levels can be divided more scientifically, which can reduce the inconvenience caused by knowledge communication.
3. We-media age has created a good external communication environment, and it prompts the interaction channel between educators and learners of Marxist philosophy to be more smooth, more accurate, and more timely. At the same time, under the background of the information age, the dissemination of all kinds of information shows explosive growth, especially in the dissemination process of Marxist philosophy; all kinds of information sources are wide; and the quality of information is also different.

In the new media age, the quality of information release is related to the feelings of information receivers. To improve the quality of information release, information publishers often have to make preparations in information selection. In particular, publishing some information on the platform that can cause a big impact on people's ideological field requires the information publisher to prepare for it [14, 15]. When publishing the information about Marxist philosophy theory, we need to consider publishing content, form, and so on. Only when these factors are fully considered can we carry out the specific dissemination of information. Otherwise, even if the relevant information is published on the platform, the actual effect obtained by the users is not obvious and cannot bring some ideological help to the receivers of information. In real life, when many information publishers publish relevant information about Marxist philosophy, they do not have a deep understanding of Marxist philosophy; many concepts have not been deeply studied; and some theoretical knowledge has not been deeply studied. This kind of seemingly unknown state leads to deviations in the understanding of Marxist philosophy among information publishers themselves because the publishers themselves do not have a comprehensive understanding of the information. It is also impossible to mine the essence of Marxist philosophy. For this reason, the credibility of the information published by the information publisher will be reduced; the attraction to the readers will be insufficient; and the interest of the readers will not be aroused, which directly affects the effective dissemination of relevant information of Marxist philosophy within social groups, that is, the quality of information dissemination. In addition, the relevant works on Marxist philosophy have great difficulty in expressing, which makes it difficult for the information publisher to understand foreign literature [16, 17]. Generally, the information publisher publishes the views of relevant Marxist philosophy in popular and understandable mass language, and there are some problems in understanding the views and concepts. In this case, the effect of theory promotion is not obvious, affecting the spread of Marxism philosophy.

However, the rich and diverse video content of Marxist philosophy poses a great challenge to its supervision and management. Because of the breakthrough of deep learning in intelligent recognition, video content recognition technology based on deep learning has gradually become the main technology in video content recognition and analysis [18, 19]. Therefore, based on deep learning, this paper studies accurate and efficient video content recognition technology by introducing an attention mechanism and making full use of the temporal features of the video.

The contribution of this paper is that an attention-mechanism-based long-term recurrent convolutional network (LRCN) model is proposed for illegal Marxist philosophy video recognition. The rest of the paper is structured as follows. In Section 2, we study the LRCN model. Attention-based LRCN model is proposed to recognize illegal Marxist philosophy videos in Section 3. Experimental results are reported in Section 4, and Section 5 gives the conclusion of this paper.

## 2. LRCN Model

In recent years, with the deepening of deep learning, breakthroughs have been made in machine translation, speech recognition, computer vision, and other fields. With the help of the study of attention characteristics of the human brain, the introduction of attention mechanism into deep learning has become a research hotspot in the field of deep learning. Similar to the human visual system, the human eye does not focus on the whole image, but instead focuses on more interesting or important areas. Although it needs to be viewed as a whole, it still scans the image in a certain order, moving from one area to another. Therefore, it is helpful to understand and analyze video content by simulating the attention characteristics of the human brain in the video content recognition method based on deep learning.

Video data is a kind of three-dimensional data, which contains not only spatial information but also temporal information. Although convolutional neural networks (CNN) can extract robust spatial features and represent the spatial information of the video, they cannot deal with the sequence problem, extract the temporal features of the video, and represent the temporal information of the video. The recognition method based on the three-dimensional convolution kernel and the recognition method based on the two-channel CNN have improved the recognition effect compared with the recognition method based on the single frame [20]. Therefore, the temporal feature of the video plays an important role in video content recognition. However, both the recognition method based on the 3D convolution kernel and the recognition method based on dual-channel CNN only consider the video content of several consecutive frames when extracting the temporal features of the video, but for long content, more video frame information needs to be used to extract the temporal features of the video in a long time range. LSTM network is a network related to the output of the current moment of the sequence and the output of the previous moment, which can remember the state information of the sequence in a long time range [21]. Integrating CNN and LSTM networks, the CNN extracts the spatial features of video, while LSTM networks extract the temporal features of video over a long period of time and make use of complementary spatial and temporal features to recognize video content, which is helpful to the understanding and analysis of video content.

LRCN model consists of two parts: spatial feature extraction and temporal feature extraction [22]. The CNN is used to extract the spatial feature vectors of original video frames and send them to temporal feature extraction. LSTM networks are used to extract temporal feature. LSTM networks extract corresponding temporal features from the input spatial feature vectors and send them to the classifier to get the final recognition results.

## 3. Attention-Mechanism-Based LRCN Model

Due to the attention characteristic of the human brain, when faced with complex and diverse video content, especially the video content related to Marxist philosophy, the manual detection method always has high accuracy compared with other video content recognition methods. Studies have shown that one of the important properties of human visual perception is that people do not process the whole image at the beginning. Instead, they selectively focus their attention on certain visual areas and combine information from different areas to construct an internal representation of the whole image, guiding human eyes to move in the image and make decisions. LRCN model adopts the structure of CNN and LSTM networks, which cannot only capture the spatial information of video content but also capture the temporal information of video content for a long time. However, the LRCN model only takes a single video frame as input at each moment, without considering the influence of the complete video sequence on video content recognition.

Venugopalan uses a codec structure to automatically generate video descriptions [23]. The encoding part extracts video features, and the decoding part generates video description. Unlike traditional video processing methods, the model takes all video frame sequences as inputs at the same time, instead of only inputting one video frame at each moment. The input of the model is defined as follows:

(1) $$\begin{array}{c} T\left(v\right)=\frac{1}{K}\sum_{i=1}^{K}v_{i}, \end{array}$$

where *v*_*i*_ represents the feature vector of the *i*-th video frame.

The model takes all video feature vectors as inputs and pays attention to the whole video sequence information at any time, but this average way makes the video lose temporal structure information, and all video frame sequences are treated equally, which makes it impossible to distinguish useful information from interference information in the whole video. For example, a video of Marxist philosophy may contain preparatory activities, Marxist philosophy, and some words, while only the content of Marxist philosophy is directly related to the theme of teaching. Therefore, when recognizing the content of the Marxist philosophy video, the model should pay more attention to the video frame sequence of teaching.

Then the attention mechanism is introduced into the model to make the model pay attention to the whole video frame sequences, especially the video frame sequences related to the teaching of Marxist philosophy, which is helpful for recognition of Marxist philosophy video content.

CNN extracts robust spatial features and obtains fixed-size feature vectors. LSTM networks recognize video content according to input feature vectors. Therefore, CNN is regarded as an encoding network and LSTM networks as an decoding network, and an attention mechanism is introduced in the decoding process to learn attention weight. So that the model's attention falls on the effective area of the whole video, and the interference of irrelevant information to the Marxist philosophy video content recognition is eliminated, so as to extract the temporal feature with attention to identify the Marxist philosophy video content.

In the decoding process, feature vectors of whole video frame sequences are weighted as the input of the LSTM network, which is shown as follows:

(2) $$\begin{array}{c} T\left(v\right)=\sum_{i=1}^{K}w_{i}^{t}v_{i}, \end{array}$$

where *w*_*i*_^*t*^ is the weight to be learned and ∑_*i*=1_^*K*^*w*_*i*_^*t*^=1. *w*_*i*_^*t*^ reflects the tightness of the feature vector of the *i*-th frame and the set of feature vectors of the whole video at time *t*. If the content of the video frame is more related to the content of the whole video, the weight of attention will be larger.

The learning of *w*_*i*_^*t*^ is related to the hidden unit state of LSTM networks at the last moment and the feature vector at the current moment, and the correlation score of *w*_*i*_^*t*^ is shown as follows:

(3) $$\begin{array}{c} s_{i}^{t}=\tanh\left(Wh_{t-1}+Av_{i}+b\right), \end{array}$$

where *h*_*t*−1_ is the state of the hidden unit at time *t* − 1, *𝕎* and *𝔸* are the weight matrix to be learned, *b* is the bias parameter, and tanh () is the activation function [24].

The LRCN model based on the attention mechanism makes the LSTM networks selectively pay attention to the effective information in the video and reduce the interference of invalid information by learning the attention weight. The structure of the LRCN model based on the attention mechanism is shown in Figure 1.

## 4. Experimental Results and Performance Analysis

### 4.1. Setup

In the LRCN model based on the attention mechanism, the process of video content recognition mainly includes four steps: video preprocessing, spatial feature extraction, attention-based temporal feature extraction, and video content prediction of illegal Marxist philosophy.

1. Video preprocessing. At first, the data set is divided into a training set and a test set. Then, FFmpeg is used to decode the raw video stream into a sequence of video frames [25]. Each type of video has a unique identifier, numbering from 0. Different identifiers represent different video categories. Since a video clip may contain hundreds of video frames, but there is a lot of redundant information between these video frames, it is necessary to extract the key frames of these video frames before the model training and divide the video content into different video clips as input of the model. The video clips divided from the same video have the same video identification. During training, every 16 frames of video content are divided into 1 video clip, and during testing, every 8 frames of video content are divided into 1 video clip, with 8 frames of the same video content between the adjacent 2 video clips.
2. Spatial feature extraction. In the LRCN model based on the attention mechanism, the video frame sequence is first input into CNN to extract the spatial feature vector. Since the feature of the fully connected layer is a high-level semantic feature, the original spatial structure information of the video content has been lost. To ensure that the subsequent LSTM networks contain more original spatial information of video content when extracting temporal features, this paper extracts the pooled feature vector corresponding to the feature graph of the last convolutional layer in the CNN as the spatial feature vector.
3. Attention-based temporal feature extraction. Since the sequence of video frames contains the temporal information of the video, the spatial feature vectors of the video are weighted and then input into the LSTM networks. The attention weight of each moment in the LSTM networks is calculated by the LSTM unit state of the last moment and the input of the current moment, and the attention-based temporal feature is extracted.
4. Video content prediction of illegal Marxist philosophy. LSTM network takes the continuous video spatial feature vectors as input, and the extracted temporal features contain not only the spatial information of video content but also the temporal information of video content. The attention-based temporal features extracted by LSTM networks at every moment are input to the classifier for prediction, and the corresponding probability output is obtained. The category corresponding to the maximum value in the output probability is selected as the input video category and compared with the preset feature library, so as to recognize the illegal Marxist philosophy video content.

### 4.2. Experimental Environment

#### 4.2.1. Data Sets

In this paper, HMDB51, UCF101, and YouTube-8M are selected as data sets used in the experiment [26]. The content of the HMDB51 data set mainly comes from movie clips, which contains 6,766 videos divided into 51 action categories. Seventy videos are selected for each category as training videos and 30 videos as test videos. The UCF101 data set is one of the most challenging video content recognition data sets so far, which contains 13,320 videos in a total of 101 video categories, including 9,537 videos as training sets and 3,783 videos as test sets. All videos are decoded by FFmpeg at 30 fps with a resolution of 320 × 240. The YouTube-8M is a large-scale dataset that contains 350000 hours of video and 2.6 billion audio/visual features. Since there are relatively few videos related to Marx's philosophy, this paper adjusts the video content to be recognized as the video content related to philosophy.

#### 4.2.2. CNN

The CNN adopts the GoogLeNet model and is pretrained on ImageNet 2012 image recognition library. ImageNet data set is currently the largest image recognition database, containing 14 million images and covering the common things in life categories. ImageNet 2012 classification data set is a subset of the ImageNet data set, selecting 1,000 categories. The video features extracted from the pretrained GoogLeNet model can effectively represent the spatial information of the video content. When training the LRCN model based on the attention mechanism, the parameters of the GoogLeNet model do not participate in the training, and the feature map of the last convolutional layer is extracted and pooled as the spatial feature of the video. The feature size is 2,048 dimensions.

#### 4.2.3. LSTM

The number of LSTM network layers is set to 1; the number of input units is 2,048; and the number of hidden units is 512. According to different data sets, the number of output units is 51 or 101. Adam optimization algorithm is used to train the LRCN model based on the attention mechanism. The initial learning rate is set to 0.001, and the maximum number of iterations is set to 20,000.

### 4.3. Performance Analysis

This paper compares the recognition accuracy of the LRCN model based on the attention mechanism with different video content recognition methods such as VWF [27], WSL-CVCR [28], and ACSL [29] on HMDB51, UCF101, and YouTube-8M data sets, respectively, and the comparison results are shown in Figure 2. The comparison methods are summarized as follows:

- VWF is a new method of human action recognition using video and Wi-Fi clues
- WSL-CVCR is a weak supervised learning framework and a new component-based video content representation method
- ACSL is an attention-based consistent semantic learning method

As can be seen from Figure 2, on the HMDB51 data set, the LRCN model based on the attention mechanism proposed in this paper focuses attention on the temporal order of video frame sequence, with higher recognition accuracy than the other three baselines. Due to the spatial features extracted by CNN, the spatial information of video content can be represented. Therefore, in the process of video content recognition, it is more important to focus the model's attention on the temporal information of video content than on the spatial information of video content. On the UCF101 data set, the proposed model uses weighted video space feature vectors as the input of the LSTM network to extract attention-based temporal features, and the recognition accuracy is high. Therefore, in the process of video content recognition, the attention characteristics of the human brain are simulated so that the model's attention falls on the effective area of the whole video, and the interference of irrelevant information is excluded, which is conducive to the understanding and analysis of video content and the improvement of recognition effect. On the YouTube-8M data set, each algorithm has achieved higher accuracy. This is because every video in the YouTube-8M data set is public, and each video has at least 1,000 frames. Although the amount of video is very large, to reduce the storage cost and computation time, Google provides precomputed and compressed features so that the model training can be completed in a day on a single computer.

The HMDB51 data set contains 51 different categories of videos, each of which contains 30 test videos. The UCF101 data set contains 101 different categories of videos, with a total of 3,783 test videos, while YouTube-8M contains more videos in different categories. To further analyze the recognition effect of the LRCN model based on the attention mechanism on each category of video content, we select 10 categories of video content from each data set for the targeted test. This paper compares the recognition accuracy of the four models in different categories of video content in HMDB51, UCF101, and YouTube-8M data sets, and the comparison results are shown in Figures 3–5, respectively.

The video content of the HMDB51 data set includes five categories: facial-related actions, facial actions related to object interaction, body-movement-related actions, body movements with objects, and human-interaction-related actions. As can be seen from the statistical results in Figure 3, compared with the other three baselines, the recognition accuracy of eight categories of the LRCN model based on the attention mechanism is higher than that of the baselines. Among them, the recognition accuracy of the LRCN model based on the attention mechanism is much higher than that of the baselines for the categories of video content such as hit, kiss, shoot gun, talk, and smoke. In this kind of video, the video content involves the human body's action interaction or the action amplitude is small, and the video content does not change much. Therefore, in the process of video content recognition, it is necessary for the model to focus on the video frame sequence related to the video theme. Meanwhile, the LRCN model based on the attention mechanism has a slightly lower recognition accuracy for stand, punch, and other categories of video content than other models, because the action of this kind of video content is ambiguous. Therefore, the LRCN model based on the attention mechanism treats video frame sequence equally, but its recognition effect is inferior to other models.

The video content of the UCF101 data set covers five categories: human movement, human-object interaction, human-human interaction, playing musical instruments, and sports. As can be seen from the statistical results in Figure 4, compared with the other three baselines, the recognition accuracy of four categories of the LRCN model based on the attention mechanism is higher than that of the baselines, and the recognition accuracy of two categories is equal to that of the other models. Hammering, tennis swing, basketball dunk, clean and jerk, and other categories are recognized more accurately by the LRCN model based on attention mechanism than by baselines, especially for hammering category videos. The recognition rate of the other three baselines is very low, and some models could not even recognize it, while the recognition accuracy of the LRCN model based on the attention mechanism is 76.51%. This type of video content is Tai Chi. Due to the small hand movements, the spatial and temporal information of video is lost during the long-term recognition of the model. However, the attention-based LRCN model can still focus the model on the video frame sequence related to the video subject during the recognition process, thus effectively recognizing the video content. Similar to the recognition effect of the HMDB51 data set, the LRCN model based on the attention mechanism is not as effective as the basic model in recognizing ambiguous video content. As can be seen from Figure 5, the accuracy of all models on all entities in the YouTube-8M data set is very high. However, for unknown labels or some special labels, the accuracy of all models is not very high.

In particular, to verify whether the videos of Marxist philosophy on the platform are illegal, we use the video lesson and teacher entities related to YouTube-8M to conduct iterative training on the proposed model, so as to verify the accuracy. As can be seen from Figure 6, with the increasing number of iterations, the LRCN model based on the attention mechanism proposed in this paper maintains high accuracy of more than 90% for the video lesson entity in the YouTube-8M data set. This shows that the current content of Marxist philosophy is mainly transmitted in the form of lessons. As can be seen from Figure 7, with the increasing number of iterations, the training effect of all models on the teacher entity in the YouTube-8M data set is not very good because it is easy to be mistaken for other roles. But, even so, with the increasing number of iterations, the accuracy of the model proposed in this paper is also improving, basically above 80%. To sum up, the model proposed in this paper has achieved high accuracy in 2,981 videos of two entities, which can accurately and timely judge whether Marxist philosophy on the platform is illegal or not, providing a good environment for the dissemination of Marxist philosophy content.

## 5. Discussion

In this paper, we analyze the dissemination of Marxist philosophical content in the public environment. Based on the research of human visual perception, we propose to simulate the attention characteristics of the human brain in the deep learning model and make the model's attention fall on the effective area of the whole video in the process of illegal Marxist philosophy video content recognition, so as to eliminate the interference of irrelevant information on video content recognition. The LRCN model based on the attention mechanism takes weighted video spatial features as input of the LSTM network and focuses on the video frames related to the video theme in the long recognition process. Through training and testing on HMDB51, UCF101, and YouTube-8M data sets, the recognition accuracy of the LRCN model based on attention mechanism in various categories of video is analyzed. However, it is necessary to enhance the affinity and pertinence of Marxist philosophy communication in the public environment.

The affinity of Marxist philosophy can enhance the attraction of Marxist philosophy, while the pertinence of Marxist philosophy can enhance the effectiveness of Marxist philosophy, solve various problems in practice, and enhance the identity of the educated. Therefore, in order to spread Marxist philosophy more widely and meaningfully, we must enhance the affinity and pertinence of the spread.

Enhancing the affinity and pertinence of the dissemination of Marxist philosophy reveals the essence of Marxist philosophy. Marxist philosophy itself is an important science with humanity, which plays an important role in promoting national economic and social development. Therefore, it is necessary to strengthen the dissemination of Marxist philosophy. To realize the goal of educating people, in the process of disseminating Marxist philosophy theory, it is necessary to transfer the humanistic care and the spirit of educating and loving. Disseminators should further highlight the humanistic nature of Marxist philosophy by enhancing affinity and pertinence, form a harmonious and close dissemination atmosphere, and constantly stimulate the enthusiasm and initiative of learning.

Enhancing the affinity and pertinence of Marxist philosophy can better understand the dialectical relationship between subject and object. The dissemination of Marxist philosophy emphasizes the equal relationship between subject and object, and the status between subject and object is interactive and equal in the dissemination of Marxist philosophy. Especially in the age of we-media, it provides an interactive platform for the dissemination of Marxist philosophy, eliminating factors such as rank and inferiority in the dissemination process. In practical interaction, if the disseminator and receiver of Marxist philosophy can have more affinity, it is bound to improve the dissemination effect of Marxist philosophy and also help realize the infiltration of theory and the output and establishment of value in the process of interaction between subject and object. To further understand the dialectical relationship between subject and object of Marxist philosophy, it is necessary to formulate practical dissemination programs according to the different characteristics and personality differences of the receivers, inspire the receivers with sincerity so that the receivers can be respected as far as possible in the whole dissemination process, and dare to interact with the disseminators, so as to imperceptibly disseminates Marxist philosophy theory in a warm and harmonious atmosphere.

Enhancing the affinity and pertinence of the dissemination of Marxist philosophy is the inevitable requirement of Marxist humanism. Under the background of the we-media age, people's values are being impacted by diversified social trends of thought, especially under the background of the market economy, people's thoughts and behaviors are changing from following traditional ideas to following the direction of fairness and equality. However, Marxist philosophy is just the value guidance to correct, solve, and adapt to the development of the times. Affinity and pertinence of Marxist philosophy are better able to respect and care for the educated, solve problems in their real lives, gradually enhance the recognition and participation in Marxist philosophy, and sublimate their values and ideal beliefs through continuous interaction with Marxist philosophy.

## Figures and Tables

**Figure 1:** Architecture of attention-mechanism-based LRCN model.

**Figure 2:** Recognition accuracy of different video content recognition methods on HMDB51, UCF101, and YouTube-8M data sets.

**Figure 3:** Recognition accuracy of 4 models in 10 actions on HMDB51 data set.

**Figure 4:** Recognition accuracy of 4 models in 10 actions on UCF101 data set.

**Figure 5:** Recognition accuracy of 4 models in 10 actions on YouTube-8M data set.

**Figure 6:** Recognition accuracy of 4 models in Video lesson entity on YouTube-8M data set.

**Figure 7:** Recognition accuracy of 4 models in Teacher entity on YouTube-8M data set.

## Data Availability

All data used to support the findings of the study are included within the paper.
